The article "Production of recombinant Entamoeba histolytica pyruvate phosphate dikinase and its application in a lateral flow dipstick test for amoebic liver abscess" was retracted in 2022. Reasons: duplicated images; concerns about the images.

# Production of recombinant *Entamoeba histolytica* pyruvate phosphate dikinase and its application in a lateral flow dipstick test for amoebic liver abscess

**DOI:** 10.1186/1471-2334-14-182

**Published:** 2014-04-04

**Authors:** Syazwan Saidin, Muhammad Hafiznur Yunus, Nor Dyana Zakaria, Khairunisak Abdul Razak, Lim Boon Huat, Nurulhasanah Othman, Rahmah Noordin

**Affiliations:** 1 Institute for Research in Molecular Medicine, Universiti Sains Malaysia, Penang 11800, Malaysia; 2 School of Materials and Mineral Resources Engineering, Engineering Campus, Universiti Sains Malaysia, 14300 Nibong Tebal, Penang, Malaysia; 3 NanoBiotechnology Research and Innovation (NanoBRI) Institute for Research in Molecular Medicine, Universiti Sains Malaysia, Penang 11800, Malaysia; 4 School of Health Sciences, Universiti Sains Malaysia, Kubang Kerian, Kelantan 16150, Malaysia

**Keywords:** *Entamoeba histolytica*, Amoebic liver abscess, Diagnosis, Recombinant pyruvate phosphate dikinase, Western blot, Lateral flow dipstick test

## Abstract

**Background:**

Amoebic liver abscess (ALA) is the most common clinical manifestation of extraintestinal amoebiasis especially in developing countries, causing up to 100 000 fatal cases annually. Accurate and early diagnosis is important to prevent the disease complications, however its diagnosis still poses many challenges due to the limitations of the available detection tools. Pyruvate phosphate dikinase (PPDK), an excretory-secretory protein of *E. histolytica*, has been reported as a potential diagnostic marker for ALA, hence it may be exploited in the development of a new test for ALA.

**Methods:**

Recombinant PPDK (rPPDK) was expressed, purified and evaluated by Western blot. In parallel, recombinant galactose-and-N-acetyl-D-galactosamine inhibitable lectin (Gal/GalNAc lectin) was produced and tested similarly. The protein identity was confirmed by analysis using MALDI-TOF/TOF. A lateral flow dipstick (LFD) test using rPPDK was subsequently developed (rPPDK-LFD) and evaluated for serodiagnosis of ALA.

**Results:**

rPPDK was expressed as soluble protein after 4 hours of induction with 1 mM isopropyl β-D-1-thiogalactopyranoside (IPTG) at 30°C. Purification using nickel-nitrilotriacetic acid (Ni-NTA) resin yielded 1.5 mg of rPPDK from 1 L of culture with estimated molecular mass of 98 kDa on SDS-PAGE. Western blots using sera from patients with ALA, healthy individuals and other diseases probed with anti-human IgG_4_-HRP showed the highest sensitivity (93.3%) and specificity (100%); as compared to blots using IgG and IgG_1_ as secondary antibodies. Moreover, rPPDK showed better specificity when compared to rGal/GalNAc lectin. In the development of the LFD test, the optimum amount of rPPDK was 0.625 μg per dipstick and the optimum working concentration of colloidal gold conjugated anti-human IgG_4_ was optical density (OD) 5 (1.7 μg of anti-human IgG_4_). Evaluation of rPPDK-LFD using ALA patients and controls serum samples showed 87% diagnostic sensitivity and 100% specificity.

**Conclusion:**

The developed rPPDK-LFD showed good potential for rapid diagnosis of ALA, and merit further multicentre validation using larger number of serum samples.

## Background

The enteric protozoan parasite, *Entamoeba histolytica* is the causative agent of amoebiasis which affects 40–50 million individuals worldwide [1]. About 10% of infected people risk developing symptomatic invasive amoebiasis namely amoebic colitis and extraintestinal amoebiasis. About 40 000 to 100 000 of fatal cases are recorded annually, most cases are due to amoebic liver abscess (ALA) which resulted from the hematogenous spread of the *E. histolytica* trophozoites from intestine to liver through the portal vein [2,3]. Other than variability in clinical manifestations [4], imaging techniques such as ultrasound, computed tomography, and magnetic resonance may not distinguish ALA from pyogenic liver abscess [5]. Therefore, serological tests are important for detection of *E. histolytica* infection to support clinical and radiological findings*.*

Currently, commercially available *E. histolytica* antibody detection assays include RIDASCREEN Entamoeba IgG ELISA (R-Biopharm AG, Darmstadt, Germany), IHA Cellognost® Amoebiasis kit (Dade Behring Marburg GmbH, Marburg, Germany) and Novagnost *Entamoeba* IgG (NovaTec Immunodiagnostica GmbH, Dietzenbach, Germany); these used complex mixture of native *E. histolytica* proteins from trophozoites [6,7]. Such tests are useful in detecting anti-*E. histolytica* antibodies in serum samples in non-endemic areas, however they often detect past infections when used in endemic areas due to the high level of background antibodies against the plethora of proteins in the native antigen [8,9]. Among the commercially available stool antigen tests, TechLab *E. histolytica* II ELISA (TechLab, Blacksburg, VA, USA) has been evaluated for detection of *E. histolytica* Gal/GalNAc lectin antigen in serum samples from patients with ALA [4,10]. However variable sensitivities have been observed depending on whether treatment had been initiated [9]. DNA-based techniques are available, however the usage is limited to reference laboratories; moreover, it requires an invasive procedure to collect the pus samples [11-13]. Therefore a convenient, rapid and sensitive serological detection test is needed to fulfil the gap in diagnosis of ALA.

Previously we have showed the promising performance of *E. histolytica* pyruvate phosphate dikinase (PPDK) as a diagnostic marker [14], thus the present study was performed to produce the recombinant protein of PPDK (rPPDK) and analyze the diagnostic sensitivity and specificity by Western blot. As a comparison, recombinant Gal/GalNAc lectin (rGal/GalNAc lectin) was also produced and similarly evaluated. Subsequently rPPDK was used in the development of lateral flow dipstick (LFD) test for the detection of specific antibodies in patients with ALA.

## Methods

### Ethics statement

The serum samples were collected from Hospital Universiti Sains Malaysia, Kubang Kerian, Kelantan, Hospital Sultanah Bahiyah, Alor Setar, Kedah and General Hospital Pulau Pinang. Serum samples from healthy volunteers and other diseases were obtained from our existing serum bank. Written informed consent for participation in the study was obtained from participants or, where participants are children, a parent or guardian. This study was approved by the Ethics Committee of the Universiti Sains Malaysia, Malaysia (ref: USMKK/PPP/JEPcm[213.3(10)]).

### Serum samples

Thirty serum samples from patients with ALA were divided into two groups namely Group A comprised 15 samples which were seropositive (for anti-*E. histolytica* antibody) and their liver abscesses were positive for *E. histolytica* DNA using real-time PCR; Group B comprised 15 samples which were seropositive but their liver abscess samples were unavailable for DNA analysis. Seropositivity was determined using RIDASCREEN *Entamoeba histolytica* IgG ELISA kit (R-Biopharm AG, Germany). Meanwhile, detection of *E. histolytica* DNA in the liver abscess aspirates was performed using real-time PCR, as published in our previous report [15]. Twenty sera from healthy individuals were used as negative control. In addition, control samples included sera from patients with other diseases (*n* = 20); i.e. toxoplasmosis (*n* = 2), malaria (*n* = 4), hydatidosis (*n* = 2), pyogenic liver abscess (*n* = 5), typhoid (*n* = 1), leptospirosis (*n* = 4) and filariasis (*n* = 2). All control sera tested negative with the above ELISA kit.

### Expression and purification of the recombinant proteins

The PPDK gene (Accession no: EHI009530) and C-terminus of Gal/GalNAc lectin gene (Accession no: AF337950) were each custom-cloned into the expression vector pET28a(+) (Novagen, Darmstadt, Germany). This vector is under control of promoter recognized by T7 RNA polymerase and contains a metal binding domain of six histidine residues for use in the affinity purification of the recombinant protein. Five microliters of each constructed plasmid was transformed into *Escherichia coli* strain BL21 (DE3) (Invitrogen, New York, USA) using CaCl_2_ method and the transformants were incubated in 200 μl of Super Optimal Broth (SOB) medium at 37°C for 1 hour prior to plating. Protein expression was performed by growing a single colony of pET28a/PPDK and pET28a/Gal-GalNAc lectin in Terrific Broth (TB) medium supplemented with 50 μg/ml of kanamycin at 37°C overnight. TB medium containing antibiotics was inoculated by overnight culture and grown at 37°C with vigorous shaking until the OD_600_ reached 0.4 to 0.6. Subsequently, the culture was induced by 1 mM IPTG (Thermo Scientific Pierce, Massachusetts, USA) for 4 hours at 30°C. To verify the presence of the histidine fusion recombinant protein, the rPPDK and rGal/GalNAc lectin protein were separated by SDS-PAGE, transferred to nitrocellulose membrane and analyzed by Western blot using anti-His conjugated to horseradish peroxidise (HRP) (Novagen, Germany) at a 1:5000 dilution. *E.coli* transformed with expression vector, pET28a(+) without insert was used as negative control.

Cells were harvested from 1 L TB liquid culture by centrifugation (10 000 *× g*, 30 min, 4°C) and the pellet were resuspended in cold lysis buffer (50 mM NaH_2_PO_4,_ 300 mM NaCl, 10 mM imidazole) at pH 8.0. Lysozyme (Amresco, Ohio, USA) at the concentration of 0.5 mg/ml was added to the suspension and incubated on ice for 30 min. The cells lysates were then disrupted by sonication (Misonix Sonicator 3000, Cole-Parmer, Illinois, USA) on ice for 3 min (30s on/30 s off). The supernatant was then treated with DNase1 (Amresco, USA) to a final concentration of 0.5 μg/ml and incubated at 4°C for 30 min followed by centrifugation at 10 000 *× g* (Avanti J-26XPi, Beckman-Coulter, California, USA) for 30 min to remove the debris. The supernatant was filtered through a 0.45 μm filter membrane (Millipore, Massachusetts, USA).

The filtered lysate of each rPPDK and rGal/GalNAc lectin proteins was purified by using nickel-nitrilotriacetic acid resin (QIAGEN GmbH, Hilden, Germany). The unpurified recombinant protein was incubated with the resin mixture at room temperature for 30 min with gentle shaking, and the resin was transferred into a column. After washing with a gradient of buffers (50 mM sodium phosphate, 500 mM sodium chloride, 20–40 mM imidazole at pH 8.0), the bound proteins was eluted with the elution buffer (50 mM sodium phosphate, 500 mM NaCl, 250 mM imidazole at pH 8). Fractions were collected at 500 μL each for up to 10–15 fractions. The purity of the protein in each fraction was determined by SDS-PAGE. Fractions with high purity proteins were pooled and concentrated using Vivaspin column with 3000 kDa cut-off (GE Healthcare, Buckinghamshire, UK). The protein concentration was determined using Bio-Rad Protein assay reagent (Bio-Rad, California, USA) and then stored at -80°C.

### Analysis of rPPDK and rGal/GalNAc lectin using MALDI-TOF/TOF

The specific protein band from SDS–PAGE gel stained with Coomassie Brilliant Blue G-250 (Bio-Rad, USA) was excised manually and destained with a commercial destaining solution (Bio-Rad, USA) at 37°C for 10 minutes; then washed with 25 mM ammonium bicarbonate (NH_4_HCO_3_, pH 7) and acetonitrile (ACN) for 10 min each. The gel plug was then reduced with 10 mM DTT and incubated at 60°C for 30 minutes, alkylated with 55 mM AAT and incubated in the dark for 60 minutes followed by digestion with 25 μl of 12.5 ng/μl trypsin (Promega, Wisconsin, USA) and incubated at 37°C for 16 h. Then, the peptides were collected into a fresh tube and the gel was further extracted using 50% ACN and 50% ACN in 0.1% TFA. The sample was then concentrated using a vacuum concentrator (Thermo Scientific Pierce, USA) until it reached half the original volume; subsequently it was freeze dried overnight (Labconco, Missouri, USA). Sample clean-up was performed using Zip-Tip columns (Millipore, USA), the peptides was then mixed with the matrix solution (a-cyano-4-hydroxy-cinnamic acid, 10.0 mg/ml, in 50% acetonitrile and 0.1% trifluoroacetic acid). Then, 0.6 μl of the mixture was spotted on a MALDI plate (three spots per sample) and allowed to dry. The sample was ran on a MALDI-TOF/TOF 5800 analyzer mass spectrometer (AB Sciex, Massachusetts, USA). One thousand shots were accumulated for MS analysis. The top fifty most intense parent ions were selected for MS/MS using air with collision energy of 2 kV and a collision gas pressure of ~ 1 × 10^-6^ Torr with 2000–3000 shots accumulated depending on the quality of the spectra. The mass spectra were searched by ProteinPilot software (AB Sciex, USA) against AmoebaDB and SwissProt using MASCOT search engine version 2.1 (Matrix Science, London, UK). The parameter search allowed for N-terminal acetylation, cysteine C-terminal carbamidomethylation and methionine oxidation. One hundred and fifty ppm and ± 0.4 Da were set for the peptide mass tolerance and fragment mass tolerance, respectively.

### Evaluation of the antigenicity of the recombinant proteins by Western blotting

The electrophoresed rPPDK and rGal/GalNAc lectin antigens from gels were transferred onto nitrocellulose (NC) membrane in alkaline transfer buffer (25 mM Tris-base, 190 mM glycine, 10% v/v methanol) using the Trans-Blot SD (Bio-Rad, USA). The membrane was then incubated in 5× Detector Block solution (KPL, Maryland, USA) for 1 h at room temperature. The membrane was then washed in TBST buffer (10 mM Tris–HCl; pH 7.5, 150 mM NaCl, 0.05% Tween-20) in 5, 10 and 15 min. Subsequently, the NC membrane was cut into multiple strips and incubated with serum samples from patients with ALA (Group A), healthy individuals and other diseases as primary antibodies at dilution 1:100 in TBST overnight at 4°C. Group B serum samples were not used since these were not from patients with PCR-proven ALA. It was important to use ‘clear-cut’ samples for proper comparison among IgG-IgG_1_- and IgG_4_-Western blots results since the assay with the higher diagnostic potential was subsequently used to develop the lateral flow test. The excess serum was removed by washing the strips with TBST.

Next, the strips were incubated with monoclonal anti-human IgG-HRP (Invitrogen, USA), IgG_1_-HRP (Invitrogen, USA) and IgG_4_-HRP (Invitrogen, USA) at dilutions of 1:6000, 1:3000 and 1:5000, respectively. The strips were washed again to remove unbound secondary antibody and subsequently developed on CL-XPosure film (Thermo Scientific Pierce, USA) using enhanced chemiluminescence (ECL) substrate system (Thermo Scientific Pierce, USA). The diagnostic sensitivity and specificity of both recombinant proteins were calculated using the formulae by Altman [16]. Sensitivity = TP/(TP + FN) × 100% and specificity = TN/(TN + FP) × 100%, where TN is the number of true negatives, TP is the number of true positives, FN is the number of false negatives, and FP is the number of false positives.

### Development of lateral flow dipstick (LFD)

**Conjugation of monoclonal mouse anti human-IgG**_**4**_** to colloidal gold**

The gold colloid was prepared using the seeding-growth method as previously described [17]. The optical density (OD) of colloidal gold particles was determined using UV–vis-NIR spectrophotometer (UV-3600, Shimadzu, Japan). First, the pH of the gold colloid was adjusted to the isoelectric point (pH 7) of the monoclonal mouse anti-human IgG_4_ antibody (Invitrogen, USA) by adding 0.2 M K_2_CO_3_. The optimum amount of anti-human IgG_4_ to be added to 10 ml of colloidal gold (OD 1.0) was 80 μg; this was obtained by observing the lowest amount of antibody that did not change colour after adding 10% NaCl. It was gently mixed and incubated for one hour at room temperature, followed by the addition of 1% bovine serum albumin (BSA) (Sigma, Missouri, USA) in water (Millipore, USA) to stabilize the mixture. The excess unconjugated antibody was removed and the remaining unbound sites on the colloidal gold were blocked by incubating with 5% BSA, then washed. The final sedimented colloidal gold conjugated IgG_4_ (at OD 20) was resuspended in 1% BSA to a final volume of 300 μl, then stored at 4°C.

### Preparation of lateral flow dipstick (rPPDK-LFD)

The rPPDK was used as the test line by jetting it linearly onto a Hi-flow Plus 90 membrane card (301 mm length) with flow rate of 90 ± 23 sec/4 cms (Milipore, USA) using IsoFlow™ Dispenser (Imagene Technology, New Hampshire, USA). The equipment was set to dispense the recombinant antigen at 0.1 μl/mm on the card. The control line comprised goat anti-mouse IgG (Invitrogen, USA) at 0.5 mg/ml. After the lined reagents have dried, the card was gently wetted with a blocking solution (Roche Diagnostics, Mannheim, Germany). After overnight drying, the membrane card was cut into 5 mm strips using Index Cutter-I (A-Point Technologies, Minnesota, USA), then stored in a dry cabinet at room temperature.

### Optimization of antigen concentration and OD of colloidal gold conjugate

Various antigen concentrations (0.7 mg/ml, 0.8 mg/ml, 0.9 mg/ml, 1.0 mg/ml, 1.25 mg/ml and 1.5 mg/ml) were tested with the initial OD of 4 to select the optimum concentration rPPDK which give the highest diagnostic sensitivity and specificity. Then, the selected rPPDK concentration was tested with various ODs of conjugated antibody, from OD 4 to 10.

### Test procedure

Serum sample was diluted 1:2 in phosphate-buffered saline (PBS, pH 7) and 30 μl placed in a well of a microtiter plate. The rPPDK-LFD was placed in the well and the sample was allowed to flow up the dipstick by capillary action. When the sample reached the top of the strip, the dipstick was dipped into another well containing 25 μl colloidal gold conjugated anti-human IgG_4_. After the line (s) was well-developed, the dipstick was dipped in another well containing PBS to wash the excess colloidal gold-conjugated IgG_4_. The result could be evaluated within 15 min; the test was recorded as ‘positive’ when two purplish red lines (control and test lines) were observed; and recorded ‘negative’ when only one purplish red line (control line) was observed. The diagnostic sensitivity and specificity of the rPPDK-LFD were determined by testing with sera of patients with ALA (Groups A and B), healthy individuals and other diseases.

## Results

### Expression and purification of the rPPDK and rGal/GalNAc lectin, and confirmation by MALDI-TOF/TOF

The optimal conditions for growth of the recombinant bacteria were at 30°C with 4 hours of post-induction with 1 mM IPTG. A satisfactory amount of soluble rPPDK, 1.5 mg PPDK per litre of culture, was obtained. SDS-PAGE analyses showed the molecular weight of the purified rPPDK and rGal/GalNAc lectin proteins were approximately 98 kDa and 53 kDa, respectively (Figures 1 and 2). The values were in an agreement with the molecular size predicted from Protparam tool [http://web.expasy.org/protparam/]. The expressions of rPPDK and rGal/GalNAc lectin proteins were further confirmed by Western blot using anti- His-HRP (Novagen, Germany) as illustrated in Figure 3. The MALDI-TOF/TOF analysis confirmed the presence of PPDK (Accession no: EHI_009530) in 98 kDa purified protein band with protein score of 465 (cut-off value > 70 indicated the significant hit), nine peptides sequences matched to the amino acid sequence and sequence coverage of 16%. Meanwhile, the result of MALDI-TOF/TOF analysis of rGal/GalNAc lectin also confirmed the presence of this protein (Accession no: EHI_006980) with protein score of 168 (cut-off value > 70 indicated the significant hit), two matched unique peptides and 6% sequence coverage. The low number of hits may be due to the fact that Gal/GalNAc lectin is a glycoprotein which is more difficult to digest using the common digestion protocol.

**Figure 1:** **SDS-PAGE analysis shows the purified rPPDK.** Lane 1: Precision Plus Protein™ Unstained Standard Marker (Bio-Rad, USA); Lane 2: Non-induced cell from pET28a/PPDK; Lane 3: Induced cell from pET28a/PPDK; Lanes 4–5: purified rPPDK protein from elution buffer (250 mM imidazole). Arrow indicates the recombinant PPDK protein (~98 kDa).

**Figure 2:** **SDS-PAGE analysis shows the purified rGal/GalNAc lectin.** Lane 1: Precision Plus Protein™ Unstained Standard Marker (Bio-Rad, USA); Lane 2: Non-induced cell from pET28a/Gal-GalNAc lectin; Lane 3: Induced cell from pET28a/Gal-GalNAc lectin; Lanes 4–5: purified rGal/GalNAc lectin protein from elution buffer (250 mM imidazole). Arrow indicates the recombinant Gal/GalNAc lectin protein (~53 kDa).

**Figure 3:** **Western blot of rPPDK and rGal/GalNAc lectin using anti-His-HRP (Novagen, Gemany).** Lane 1: Precision Plus Protein™ Unstained Standard Marker (Bio-Rad, USA); Lanes 2 and 4: *E.coli* whole cells transformed with pET28a(+) vector as a control; Lane 3: *E.coli* whole cells expressed rPPDK; Lane 5: *E.coli* whole cells expressed rGal/GalNAc lectin.

### Evaluation of the rPPDK and rGal/GalNAc lectin protein via Western blot

Table 1 summarizes the Western blot results of rPPDK and rGal/GalNAc lectin using serum samples from patients with ALA (*n* = 15), healthy individuals (*n* = 20) and patients with other diseases (*n* = 20). Using IgG, IgG_1_ and IgG_4_ as secondary antibodies, anti-PPDK antibodies were detected in 13 (86.7%), 12 (80%) and 14 (93.3%) of 15 ALA patients, while anti-Gal/GalNAc lectin antibodies were detected in 13 (86.7%), 12 (80%) and 14 (93.3%) of 15 ALA patients. The rPPDK showed 97.5%, 97.5% and 100% specificities while rGal/GalNAc lectin showed 97.5%, 87.5% and 95.0% specificities when probed with IgG, IgG_1_ and IgG_4,_ respectively. Therefore, the rPPDK probed with mouse anti-human IgG_4_ was chosen for development of lateral flow dipstick as it showed the highest diagnostic sensitivity and specificity. Figures 4 and 5 illustrated the representative IgG, IgG_1_ and IgG_4_ blots of rPPDK and rGal/GalNAc lectin protein probed with human serum samples.

**Table 1:** **Reactivity of the rPPDK and rGal/GalNAc lectin from blots probed with anti-human IgG-HRP, IgG**_**1**_**-HRP and IgG**_**4**_**-HRP**

**Recombinant proteins**	**Secondary conjugate peroxidase**	**Serum from patients with ALA (Group A)**	**Serum from healthy individuals and patients with other diseases**
Pyruvate phosphate dikinase (rPPDK)	IgG	86.7% (13/15)	97.5% (39/40)
	IgG_1_	80.0% (12/15)	97.5% (39/40)
	IgG_4_	93.3% (14/15)	100% (40/40)
Gal/GalNAc lectin	IgG	86.7% (13/15)	97.5% (39/40)
(rGal/GalNAc lectin)			
	IgG_1_	80.0% (12/15)	87.5% (35/40)
	IgG_4_	93.3% (14/15)	95.0% (38/40)

**Figure 4:** **Representative IgG, IgG**_**1**_**and IgG**_**4**_**blots of rPPDK probed with human serum samples.** Lane 1: Precision Plus Protein™ Unstained Standard Marker (Bio-Rad, USA); Lanes 2 to 3: individual serum samples from patients with ALA probed with IgG; Lanes 4 to 5: individual serum samples probed from patients with ALA probed with IgG_1_, Lanes 6 to7: individual serum samples from patient with ALA probed with IgG_4_; Lanes 8, 10 and 12: negative serum samples from healthy individuals probed with IgG, IgG_1_ and IgG_4_, respectively; Lanes 9, 11 and 13: negative serum samples from other disease probed with IgG, IgG_1_ and IgG_4,_ respectively.

**Figure 5:** **Representative IgG, IgG**_**1**_**and IgG**_**4**_**blots of rGal/GalNAc lectin probed with human serum samples.** Lane 1: Precision Plus Protein™ Unstained Standard Marker (Bio-Rad, USA); Lanes 2 to 3: individual serum samples from patients with ALA probed with IgG; Lanes 4 to 5: individual serum samples probed from patients with ALA probed with IgG_1_, Lanes 6 to7: individual serum samples from patient with ALA probed with IgG_4_; Lanes 8, 10 and 12: negative serum samples from healthy individuals probed with IgG, IgG_1_ and IgG_4_, respectively; Lanes 9, 11 and 13: negative serum samples from other disease probed with IgG, IgG_1_ and IgG_4,_ respectively.

### Optimum antigen concentration and OD of colloidal gold conjugate

The optimum concentration of rPPDK for the test line was 1.25 mg/ml or 0.125 μg per mm of the membrane card, thus each dipstick contains 0.625 μg rPPDK. The optimum working concentration for colloidal gold conjugated anti-human IgG_4_ was OD 5. At 25 μl of conjugated antibody used per dipstick, this corresponded to approximately 1.7 μg of anti-human IgG_4_ per test.

### Sensitivity and specificity of rPPDK-LFD

The results of the diagnostic evaluation of rPPDK-LFD test are summarized in Table 2. Twenty six serum samples from 30 patients with ALA were tested positive with rPPDK-LFD with 87% sensitivity and 100% specificity. Four samples from Groups A and B ALA patients were found to be negative; one from Group A and 3 from Group B. From Group A, the same sample was also negative by IgG_4_-Western blot. No cross reactivity was observed from the negative samples. Representative images of rPPDK-LFD tested with various serum samples are shown in Figure 6.

**Table 2:** Sensitivity and specificity of the lateral flow dipstick for detection of anti-PPDK antibodies in serum samples

**Lateral flow dipstick test result**	**No. of serum samples that had been tested for the presence of anti-PPDK antibodies**		
	**Positive**	**Negative**	**Total**
Positive	26^*a+b*^	0	26
	(87%)*		
Negative	4^*a+b*^	40^*c+d*^	44
		(100%) **	
Total	30	40	70

^*a*^Group A sera : Seropositive and *E. histolytica* DNA detected in patients’ liver abscess samples.

^*b*^Group B: sera Seropositive and liver abscess samples non-available for DNA analysis.

^*c*^Healthy individuals, Seronegative.

^*d*^Other diseases: Seronegative (i.e.: pyogenic liver abscess, malaria, toxoplasmosis, leptospirosis, hydatidosis, filariasis and typhoid).

*Sensitivity tested with 30 sera from patients with ALA (Groups A and B).

**Specificity tested with 40 sera from healthy individuals and patients with other diseases.

**Figure 6:** **Representative rPPDK-LFD strips tested with serum samples.** Lanes 1–3: Lateral flow test strips reacted with serum samples from patients with ALA; Lane 4: strips reacted with serum from healthy individual; Lanes 5–6: strips reacted with serum samples from other diseases (i.e. malaria and pyogenic liver abscess), C: control line; T: test line.

## Discussion

*E. histolytica* remains a public health threat in many parts of the world, especially in the low-resource developing countries, and has re-emerged in some previously dormant areas [18]. The most common extraintestinal manifestation of this infection is ALA, which is associated with significant morbidity and mortality [19]. Serodiagnosis is widely used for detection of ALA, and several assays for the detection of anti-*E. histolytica* antibodies have been developed. These include indirect hemagglutination (IHA), latex agglutination, counter-immunoelectrophoresis (CIE), amoebic gel diffusion test, indirect immunofluorescence assay (IFA) and ELISA. Although ELISA is the most promising in terms of sensitivity [4,8,20], it is usually based on detection of long-lived IgG antibodies which causes difficulty to distinguish current from past infections especially in endemic settings [21]. In addition, most of the commercial diagnostic tests utilize *E. histolytica* crude soluble antigen, thus cross reactions with antibodies to other infections may be an issue [4,10]. It is also difficult and time consuming to maintain *E. histolytica* trophozoites in culture, to propagate large amounts of the parasite and consistently produce high quality antigen [7]. Therefore, there is a need to improve the diagnosis of ALA by using recombinant proteins which are known to be more specific and reproducible. Recombinant proteins for *E. histolytica* antibody detection assays have been reported, such as 70 kDa rPGM protein, Gal/GalNAc-specific lectin and serine-rich *E.histolytica* protein; they showed sensitivities and specificities ranging from 80% to 100% when tested using ELISA [7,22-24]. In addition, a study using recombinant antigen to Gal/GalNAc lectin (termed as LecA), in a flowthrough rapid test was reported to be 97% sensitive and 100% specific for diagnosis of ALA [25]. However there is still a need to convert the recombinant antigen-based test into a lateral flow immunochromatography test which is rapid, easy to perform and interpret, and can be transported at room temperature.

In a previous study by our group, PPDK of *E. histolytica*, an enzyme involved in the protozoan glycolytic pathway, was found to be useful for diagnosis of ALA with 82% sensitivity and 100% specificity by Western blot [14,26]. Thus in this study, PPDK was produced as a recombinant protein by employing pET expression vector system in *E. coli*, and the optimized expression conditions produced 1.5 mg PPDK per litre of culture. Western blots performed using serum samples of ALA patients and controls showed that detection of anti-amoebic IgG_4_ antibody in samples from patients with ALA exhibited the highest sensitivity and specificity, as compared to detection of IgG and IgG_1_. In addition, comparison was made between rPPDK and the previously reported rGal/GalNAc lectin. The latter was a C-terminal segment of the full protein, which was reported to be highly sensitive and specific for detection of ALA [27]. In IgG_4_ assay, the diagnostic sensitivities of both molecules were similar, however rPPDK demonstrated better specificity. Thereafter, the rPPDK was used in the development of an IgG_4_ lateral flow test in a dipstick format. The optimized parameters of the rPPDK-LFD test and colloidal gold conjugated anti-human IgG_4_ showed diagnostic sensitivity of 87% and specificity of 100%. With regard to the test sensitivity, 3 of 15 samples from Group B of the ALA patients were not reactive. Some possible reasons could be due to extremely low or lack of anti-PPDK antibodies in these samples; possibly these were from patients with non-active infection. There was no cross reactivity with serum samples from healthy individuals and other diseases, suggesting that this assay is highly specific for detection of ALA. Further multicentre validation studies are thus warranted using a larger number of serum samples from different geographical regions, inclusion of serum samples from patients infected with *Schistosoma* and *Fasciola hepatica*, patients with other extraintestinal amoebiasis, as well as sera from pre- and post-treatment patients. When validated, the rapid test would be useful for disease diagnosis and control; and for epidemiological studies.

Currently recombinant proteins such as rPPDK and rGal/GalNAc lectin may not be easily accessible to scientists and diagnostic laboratories as compared to crude extract of *E. histolytica* from axenic culture of the parasite. However, since recombinant proteins hold promise of greater diagnostic specificity, it is imperative that the recombinant antigen-based tests should be made commercially available.

## Conclusion

The rPPDK-LFD described in this study showed promise as a rapid diagnostic test for patients suspected of ALA. It fulfills WHO ASSURED criteria [28,29] for tests that address disease control needs i.e. specific, sensitive, simple and convenient, and results that can be rapidly read by naked eye. The test can be used in clinical laboratories which lack specialized equipments or skilled personnel; or where the low number and frequency of patients do not justify purchase of ELISA kits.

### Consent

Written informed consents were obtained from the patients for publication of this report.

## Competing interest

RN, LBH, NHO are named as inventors in a related patent application made by Universiti Sains Malaysia, entitled “Diagnosis of *Entamoeba histolytica*”, which was filed in Malaysia (PI 2011003202) and PCT (PCT/MY2011/000172).

## Author’s contributions

Conceived and designed the experiments: RN, SS. Performed the experiments: SS, DZ, MHY. Analyzed and interpreted the data: SS, RN. Contributed reagents/materials/analysis tools: LBH, NHO, KAR. Wrote the paper: SS, RN, NHO, DZ. All authors participated in editing the paper. All authors read and approved the final manuscript.

## Pre-publication history

The pre-publication history for this paper can be accessed here:

http://www.biomedcentral.com/1471-2334/14/182/prepub
